RETRACTED

# PM2.5 Exposure Induces Lung Injury and Fibrosis by Regulating Ferroptosis *via* TGF-*β* Signaling

**DOI:** 10.1155/2022/7098463

**Published:** 2022-09-27

**Authors:** Li Guo, Shuping Bai, Shaohua Ding, Ling Zhao, Shanqi Xu, Xiaohong Wang

**Affiliations:** Department of Respiratory Medicine, Harbin Medical University Cancer Hospital, No. 150 Haping Road, Harbin 150081, China

## Abstract

**Background:**

Lung fibrosis is a severe lung disorder featured by chronic nonspecific inflammation of the interstitial lung and deposition of collagen, leading to lung dysfunction. It has been identified that ferroptosis is involved in the progression of lung injury. Particulate matter (PM2.5) is reported to be correlated with the incidence of pulmonary fibrosis. However, mechanisms underlying ferroptosis in PM2.5-related lung fibrosis is unclear. In this study, we aimed to explore the effect of PM2.5 on ferroptosis in lung fibrosis and the related molecular mechanisms.

**Methods:**

PM2.5-treated mouse model and cell model were established. Fibrosis and tissue damage were measured by Masson's trichrome staining and HE staining. Fibrosis biomarkers, such as *α*-SMA, collagen I, and collagen III, were examined by histological analysis. The ferroptosis phenotypes, including the levels of iron, Fe^2+^, MDA, and GSH, were measured by commercial kits. ROS generation was checked by DCFH-DA. The oxidative stress indicators, 3-nitro-L-tyrosine (3′-NT), 4-HNE, and protein carbonyl, were checked by enzyme linked immunosorbent assay (ELISA). The thiobarbituric acid reactive substances (TBARS) and GSH/GSSG ratio were assessed by TBARS assay kit and GSH/GSSG assay kit, respectively. TGF-*β* signaling was detected by Western blotting.

**Results:**

PM2.5 induced the lung injury and fibrosis in the mice model, along with elevated expression of fibrosis markers. PM2.5 enhanced oxidative stress in the lung of the mice. The SOD2 expression was reduced, and NRF2 expression was enhanced in the mice by the treatment with PM2.5. PM2.5 triggered ferroptosis, manifested as suppressed expression of GPX4 and SLC7A11, decreased levels of iron, Fe^2+^, and MDA, and increased GSH level in mouse model and cell model. The TGF-*β* and Smad3 signaling was inhibited by PM2.5. ROS inhibitor NAC reversed PM2.5-regulated ROS and ferroptosis in primary mouse lung epithelial cells.

**Conclusions:**

Therefore, we concluded that PM2.5 exposure induced lung injury and fibrosis by inducing ferroptosis *via* TGF-*β* signaling.

## 1. Introduction

Pulmonary fibrosis serves as a prevalent interstitial lung disorder featured by chronic nonspecific inflammation of the interstitial lung and deposition of collagen, resulting in lung function impairment, and severely impaired the health and life quality of patients [1]. Unlike other kinds of lung disorders, the mechanisms of the progression of pulmonary fibrosis are still unclear [2]. Pulmonary fibrosis presents a high mortality rate and has been identified as a “tumor-like disease” [3]. The recently approved treatments for pulmonary fibrosis, such as nintedanib and pirfenidone, are indicated to repress the event of lung dysfunction [4, 5]. However, no effective strategy is currently available to improve the survival rate of patients with pulmonary fibrosis [4, 5]. Therefore, it is imperative to explore the mechanisms for prevention and treatment of pulmonary fibrosis.

RETRACTED

Recently, the frequency of pulmonary fibrosis has expanded with the growing hardness of air pollution [6]. Epidemiological investigations have revealed that the development in the incidence of pulmonary fibrosis is correlated with progressing delicate particulate matter (PM2.5, aerodynamic diameter ≤ 2.5 *μ*m) levels in the atmosphere [7]. Due to its small diameter, PM2.5 can quickly enter the alveoli or even the blood after being breathed. PM2.5 can destroy antioxidant proteins by absorbing toxic ingredients and induce injury by elevating reactive oxygen species (ROS) level, which eliminates the functions of the alveolar epithelial cells [8]. It has been reported that PM2.5 can lead to mitochondrial and DNA damage and promote autophagy of alveolar epithelial cells [9]. PM2.5 contributes to pulmonary fibrosis in mice through ROS/AKT signaling [10]. However, the understanding of the function of PM2.5 in the regulation of pulmonary fibrosis remains limited.

Ferroptosis is a newly identified programed cell death that characterized by abnormal iron metabolism, lipid metabolism, oxidative stress, and glutathione (GSH) [11]. Increasing evidence has demonstrated that ferroptosis is correlated with various diseases, including cancer, cardiovascular diseases, and neurodegenerative diseases [12–14]. Besides, previous study has identified that ferroptosis participate in the progression of lung injury [15, 16]. Noteworthy, PM2.5 induces injury of endothelial cells through triggering ferroptosis, manifested by abnormal intracellular iron content, ROS accumulation, and lipid peroxidation [17].

Transforming growth factor (TGF)-*β* is a critical regulator that participate in numerous biological processes such as tissue regeneration, development, tumorigenesis, and immune responses [18, 19]. Studies on multiple mouse models have indicated that TGF-*β* is necessary for organogenesis and homeostasis of lung [20, 21]. TGF-*β* modulates epithelial cell growth, cell differentiation, extracellular matrix remodeling, and fibroblast activation [22]. Treatment with TGF-*β*1 suppressed expression of System xc, the critical regulator of ferroptosis, in hepatocellular carcinoma cells through regulating Smad3 [23].

RETRACTED

This study is aimed at exploring the effect of PM2.5 on lung fibrosis and the related mechanism. We identified the significant function of PM2.5 in the regulation of lung fibrosis and ferroptosis by modulating TGF-*β* signaling.

## 2. Materials and Methods

### 2.1. Cell Culture

The human normal lung epithelial cell line BEAS-2B and non-small-cell lung cancer cell line A549 were purchased from Shanghai Cell Bank of Chinese Academy of Science. The primary mouse alveolar epithelial cells (AECs) were isolated from C57BL/6J mouse following a previously reported procedure [24]. In brief, the lung tissues were isolated from mouse and digested by dispase (Sigma, USA) and collagenase (Sigma) at 37°C for 30 minutes. The cell suspension was then probed by antibodies against EPCAM (eBioscience, USA), CD24, SFTPC, CD31, CD34, and CD45. The AEC2 cell population was sorted by flow cytometry as CD24^−^ SFTPC^+^ subset, apart from the EPCAM^+^CD31^−^CD34^−^CD45^−^ subset of epithelial cell populations. The obtained AECs were then cultured in Matrigel-coated 6-well plate (Corning) and bronchial epithelial cell growth medium (BEGM) that contains 1% FBS (Gibco, USA), 50 ng/mL FGF, and 30 ng/ml HGF (Sigma).

### 2.2. Animal Model

All animal experiments were authorized by the Ethics Committee of the Animal Experimental Center of Harbin Medical University Cancer Hospital (approval No. 2021-0031). Female C57BL/6J mice aged 8-weeks old were brought from Charles River Laboratory (USA), and randomly divided into three groups, including the control group of which the mice were treated with standard reference materials (SRMs), and the PM 2.5 groups of which the mice were treated with PM 2.5 for 15 or 30 days, respectively. To establish PM2.5 injury, each mouse was intratracheally instilled with 50 *μ*g PM2.5 every 5 days in 30 days. The PM 2.5 was purchased from the National Institute for Standards and Technology (NIST) (USA).

### 2.3. Histological Analysis

The lung tissues of mice were collected, fixed in paraformaldehyde, embedded by paraffin, and sectioned into 5 *μ*m slices. The lung injury in tissue samples were checked by H&E staining (Thermo, USA). The fibrosis of lung tissues was assessed by Masson's trichrome (Thermo, USA) following the manufacturer's instruction.

For immunohistochemical evaluation of collagen I, collagen III, and *α*-SMA levels, the slices were processed with antigen retrieval, then the endogenous peroxidase was inactivated by 3% H_2_O_2_. After that, the samples were incubated with specific primary antibodies against collagen I, collagen III, and *α*-SMA (Abcam, USA) at 4°C overnight. Next day, the samples were hatched with biotin-labeled secondary antibodies, followed by visualization by DAB staining kit (Beyotime, China).

RETRACTED

### 2.4. Reactive Oxygen Species Detection

To determine the ROS level, the lung tissues were digested to generate cell suspension as was mentioned above. The ROS level was determined by DCFH-DA staining (Thermo) in accordance with the manufacturer's instruction. In brief, the cell suspension was mixed with diluted DCFH-DA reagent (10 *μ*mol/l) and reacted at 37°C for 30 minutes. The cells were then detected by flow cytometry (BD Biosciences, USA).

### 2.5. Determination of Oxidative Stress and Ferroptosis Biomarkers

The levels of 3-nitro-L-tyrosine (3′-NT), 4-HNE, and protein carbonyl were checked by enzyme-linked immunosorbent assay (ELISA) using commercial kits following the manufacturer's instruction. The thiobarbituric acid reactive substances (TBARS) and GSH/GSSG ratio were assessed by TBARS assay kit (Abnova, USA) and GSH/GSSG assay kit (Abcam), respectively. The levels of iron, Fe2+, and MDA were measured by the related kit (Abcam, USA).

### 2.6. Western Blotting

Total proteins were extracted from lung tissues or cells by using an ice-cold RIPA lysis buffer (Thermo) that contains protease inhibitors (Thermo). Protein concentration was determined by a BCA Protein Assay Kit (Thermo). Equal amounts of proteins were divided by SDS–PAGE and blotted to nitrocellulose membrane, followed by block with 5% skim milk. The blots were then hatched with primary antibodies against TGF-beta1 (Proteintech, China), smad3 (Abcam, USA), TET2 (Abcam, USA), GPX4 (Abcam, USA), SLC7A11 (Abcam, USA), and tubulin (Abcam, USA) at 4°C overnight. Proteins were then visualized with corresponding horseradish peroxidase- (HRP-) conjugated secondary antibodies and ECL reagents (Millipore, USA) on a gel image system. The intensity of protein bands was quantified by Image J software.

### 2.7. Cell Viability

The cell viability was determined by cell counting kit-8 (CCK-8) (Beyotime, China) in line with the manufacturer's protocols. In short, the A549 or AECs were seeded in 96-well plates at a density of 5,000 cells per well and incubated for 24, 48, and 72 hours, At the end time points, CCK-8 reagent (20 *μ*l) was added into each well and incubated for another 2 hours. The optical density at 450 nm was assessed by a microplate reader (Thermo).

### 2.8. Detection of 5hmC Level

The levels of 5hmC in lung tissues and AECs were measured by ELISA assay kit following the manufacturer's description.

RETRACTED

### 2.9. Statistics

Data in this study are shown as mean ± SD and analyzed by GraphPad Prism 6 (USA) software and SPSS 20.0 software. Student's *t*-test or one-way analyses of variance (ANOVA) was used to compare differences between two or more groups if they followed a normal distribution; otherwise, the nonparametric Mann–Whitney test was adopted. Statistically significant data are defined as ^∗^*p* < 0.05.

## 3. Results

### 3.1. PM2.5 Promotes Lung Fibrosis in Mice

To decipher the role of PM2.5 in the regulation of lung fibrosis, the mice were treated with PM2.5. H&E staining showed that the treatment of PM2.5 induced the lung injury in the mice (Figure 1(a)). Masson staining revealed that the lung fibrosis was enhanced by the treatment of PM2.5 in the mice (Figure 1(b)). Meanwhile, the fibrosis markers, such as *α*-SMA, collagen I, and collagen III, were promoted by the treatment of PM2.5 in the mice (Figure 1(c)).

### 3.2. PM2.5 Enhances Ferroptosis in the Lung of the Mice

We then evaluated the function of PM2.5 in the modulation of ferroptosis in the mice. We found that the expression of ferroptosis negative markers, such as GPX4 and SLC7A11, was repressed by PM2.5 in the lung tissues of the mice (Figure 2(a)). The treatment of PM2.5 induced the levels of iron, Fe^2+^, and MDA but reduced the GSH levels in the model (Figures 2(b)–2(e)).

We observed that the treatment of PM2.5 promoted the levels of ROS in the mice (Figure S1A). The levels of 3′-NT, 4-HNE, TBARS, protein carbonyl, and GSH/GSSG ratio were enhanced by the treatment of PM2.5 in the mice (Figure S1B). The SOD2 expression was reduced, and NRF2 expression was enhanced by the treatment of PM2.5 in the mice (Figure S1C).

### 3.3. PM2.5 Increases TGF-beta1/smad3 Expression and Decreases TET2 and 5hmC Expression in the Lung of the Mice

Next, we explored the potential mechanism of PM2.5-mediated lung fibrosis and oxidative stress in the mice. We observed that the TGF-*β* and Smad3 expression was enhanced, and TET2 expression was reduced by the treatment of PM2.5 in the mice (Figures 3(a) and 3(b)). Consistently, the levels of 5hmC were induced by the treatment of PM2.5 in the mice (Figure 3(c)).

### 3.4. PM2.5 Promotes Ferroptosis Primary Mouse Lung Epithelial Cells

Then, we evaluated the effect of PM2.5 on ferroptosis primary mouse lung epithelial cells. We found that the treatment of PM2.5 slightly affected the cell viability of A549 cells and primary mouse lung epithelial cells (Figures 4(a) and 4(c)). Significantly, the levels of ROS were induced by the treatment of PM2.5 in A549 cells and primary mouse lung epithelial cells (Figures 4(b) and 4(d)). Moreover, the expression of ferroptosis negative markers, such as GPX4 and SLC7A11, were inhibited by PM2.5 in primary mouse lung epithelial cells (Figure 4(e)). The treatment of PM2.5 enhanced the levels of iron, Fe^2+^, and MDA but decreased the GSH levels in the model (Figures 4(f)–4(i)).

RETRACTED

### 3.5. PM2.5 Increases TGF-beta1/smad3 Expression and Decreases TET2 and 5hmC Expression in Primary Mouse Lung Epithelial Cells

Next, we observed that the treatment of PM2.5 increased TGF-*β* and Smad3 expression and decreased TET2 expression in primary mouse lung epithelial cells (Figures 5(a) and 5(b)). Meanwhile, the levels of 5hmC were promoted by the treatment of PM2.5 in primary mouse lung epithelial cells (Figure 5(c)).

### 3.6. NAC Reverses PM2.5-Regulated ROS in Primary Mouse Lung Epithelial Cells

We then assessed the effect of ROS inhibitor NAC on PM2.5-mediated ROS levels in primary mouse lung epithelial cells. We observed that the levels of ROS were increased by PM2.5 and decreased by NAC in primary mouse lung epithelial cells, in which NAC was able to reverse the effect of PM2.5 (Figure 6(a)). Meanwhile, the treatment of PM2.5 increased TGF-*β* and Smad3 expression and decreased TET2 expression, but NAC presented reversed function in primary mouse lung epithelial cells (Figures 6(b) and 6(c)). In addition, the treatment of PM2.5 induced the levels of 5hmC, while the treatment of NAC reversed the effect in primary mouse lung epithelial cells (Figure 6(d)). Moreover, the PM2.5-induced ferroptosis phenotypes was reversed by the treatment of NAC in primary mouse lung epithelial cells (Figures 6(e)–6(i)).

## 4. Discussion

Lung fibrosis serves as a severe lung disorder featured by chronic nonspecific inflammation of the interstitial lung and deposition of collagen, leading to lung dysfunction, which is closely associated with air pollution. PM2.5 has been identified as a challenging environmental problem, but the understanding of the function of PM2.5 in the regulation of lung fibrosis remains limited. Here, we discovered the crucial effect of PM2.5 on oxidative stress in lung fibrosis.

The previous studies have reported the correlation of PM2.5 with lung fibrosis. It has been reported that small GTPase RAB6 deficiency contributes to alveolar progenitor cell renewal and represses PM2.5-related lung fibrosis [25]. Adipose mesenchymal stem cell-derived extracellular vesicles relieve PM2.5-stimulated lung fibrosis [26]. DNA repair enzyme OGG1 attenuates PM2.5-associated lung fibrosis and enhances alveolar progenitor cell renewal [27]. PM2.5 causes vascular remodeling, lung inflammation, and exacerbates transition of left ventricular failure to right ventricular hypertrophy [28]. Consistent with previous studies, in this work, we found that the treatment of PM2.5 induced the lung injury in the mice. The lung fibrosis was enhanced by the treatment of PM2.5 in the mice. Meanwhile, the fibrosis markers, such as *α*-SMA, collagen I, and collagen III, were promoted by the treatment of PM2.5 in the mice. PM2.5 elevated the level of ROS in the mice lung tissue. Besides, the levels of 3′-NT, 4-HNE, TBARS, protein carbonyl, GSH/GSSG ratio, and the oxidative response biomarkers were enhanced by the treatment of PM2.5 in the mice. The SOD2 expression was reduced, and NRF2 expression was enhanced by the treatment of PM2.5 in the mice. These data present an innovative role of PM2.5 in the promotion of lung fibrosis and oxidative stress, providing crucial evidence for the important function of PM2.5 in lung injury.

RETRACTED

Moreover, it has been identified that oxidative stress plays a crucial role in the modulation of lung fibrosis. Pterostilbene reduces LPS-induced pulmonary fibrosis through inhibiting apoptosis, inflammation, and oxidative stress [29]. SIRT3 deficiency contributes to lung fibrosis by inducing mitochondrial DNA damage and apoptosis of alveolar epithelial cells [30]. GHK-Cu attenuates bleomycin-induced pulmonary fibrosis by anti-inflammation and antioxidative stress signaling [31]. Diosmin relieves lung fibrosis by targeting oxidative stress in mice [32]. Meanwhile, the function of TGF-*β* in the progression of lung fibrosis has been reported. It has been reported that curdione attenuates bleomycin-stimulated lung fibrosis *via* inhibiting TGF-*β*-related fibroblast to myofibroblast differentiation [33]. Biochanin-A suppresses lung fibrosis by repressing the TGF-*β*-mediated collagen deposition, myofibroblasts differentiation, and EMT [34]. Paeoniflorin relieves TGF-*β*-mediated EMT by Smad signaling in lung fibrosis [35]. In the present study, we found that the TGF-*β* and Smad3 expression was enhanced, and TET2 expression was reduced by the treatment of PM2.5 both in vitro and in vivo. The levels of ROS were induced by the treatment of PM2.5 in A549 cells and primary mouse lung epithelial cells. Besides, ROS inhibitor NAC reversed PM2.5-regulated ROS in primary mouse lung epithelial cells. These findings provide crucial evidence of the crucial function of ROS and TGF-*β* signaling in PM2.5-mediated lung fibrosis. Nevertheless, the modulation of TGF-*β* by PM2.5 treatment needs further study with cellular experiments. Other potential mechanisms in the regulation of PM2.5-regulated lung tissue ferroptosis should be further explored.

In conclusion, we discovered that PM2.5 exposure induced lung injury and fibrosis by regulating oxidative stress and TGF-*β* signaling. Our finding provides new insight into the mechanism by which PM2.5 regulates lung injury and fibrosis by oxidative stress and TGF-*β* signaling.

RETRACTED

## Figures and Tables

**Figure 1:** PM2.5 promotes lung fibrosis in mice. (a–c) The mice were treated with PM2.5 for 15 days or 30 days. (a) The lung injury was measured by H&E staining. (b) The lung fibrosis was detected by Masson staining. (c) The levels of *α*-SMA, collagen I, and collagen III were analyzed by IHC staining.

**Figure 2:** PM2.5 enhances ferroptosis in the lung of the mice. (a–e) The mice were treated with PM2.5 for 15 days or 30 days. (a) The expression of GPX4 and SLC7A11 was measured by Western blot. (b–e) The levels of iron, Fe^2+^, MDA, and GSH were detected in the mice. ^∗∗^*p* < 0.01.

**Figure 3:** PM2.5 increases TGF-beta1/smad3 expression and decreases TET2 and 5hmC expression in lung of the mice. (a–c) The mice were treated with PM2.5 for 15 days or 30 days. (a, b) The expression of TGF-*β*, Smad3, and TET2 was analyzed by Western blot analysis. (c) The levels of 5hmC were examined by ELISA assays. ^∗∗^*p* < 0.01.

**Figure 4:** PM2.5 promotes ferroptosis in primary mouse lung epithelial cells. (a, b) The A549 cells were treated with PM2.5 at the indicated doses. (a) The cell viability was measured by CCK-8 assays. (b) The ROS levels of were analyzed by flow cytometry analysis. (c–i) The primary mouse lung epithelial cells were treated with PM2.5 at the indicated doses. (c) The cell viability was measured by CCK-8 assays. (d) The ROS levels were analyzed by flow cytometry analysis in the cells. (e) The expression of GPX4 and SLC7A11 was measured by Western blot. (f–i) The levels of iron, Fe^2+^, MDA, and GSH were detected in the cells. ^∗∗^*p* < 0.01.

**Figure 5:** PM2.5 increases TGF-beta1/smad3 expression and decreases TET2 and 5hmC expression in primary mouse lung epithelial cells. (a–c) The primary mouse lung epithelial cells were treated with PM2.5 at the indicated doses. (a, b) The expression of TGF-*β*, Smad3, and TET2 was analyzed by Western blot analysis. (c) The levels of 5hmC were examined by ELISA assays. ^∗∗^*p* < 0.01.

**Figure 6:** NAC reverses PM2.5-regulated ferroptosis in primary mouse lung epithelial cells. (a–i) The primary mouse lung epithelial cells were treated with PM2.5 or cotreated with NAC. (a) The ROS levels of were analyzed by flow cytometry analysis. (b, c) The expression of TGF-*β*, Smad3, and TET2 was analyzed by Western blot analysis. (d) The levels of 5hmC were examined by ELISA assays. (e) The expression of GPX4 and SLC7A11 was measured by Western blot. (f–i) The levels of iron, Fe^2+^, MDA, and GSH were detected in the cells. ^∗∗^*p* < 0.01.

RETRACTED

## Data Availability

All data generated or analyzed during this study are included in this published article.

## Supplementary Materials

Supplementary Materials Figure S1: PM2.5 enhances oxidative stress in the lung of the mice. (A–C) The mice were treated with PM2.5 for 15 days or 30 days. A. The ROS levels of were analyzed by flow cytometry analysis in the mice. B. The levels of 3'-NT, 4-HNE, TBARS, protein carbonyl, and GSH/GSSG ratio were detected in the mice. C. The expression of SOD2 and NRF2 was analyzed by Western blot analysis. ^∗∗^*p* < 0.01.
